RETRACTED

# A Secure Private Cloud Storage Platform for English Education Resources Based on IoT Technology

**DOI:** 10.1155/2022/8453470

**Published:** 2022-06-14

**Authors:** Wei Li, Ying Guo

**Affiliations:** School of Foreign Studies, Tangshan Normal University, Tangshan Hebei 063000, China

## Abstract

The contemporary ubiquitous “cloud” network knowledge and information resources, as well as ecological pedagogy theory, have enlarged teaching research's perspective, widened teaching research's innovation area, and created practical options for English classroom reform. Cloud education relies on the Internet of Things, cloud computing, and big data to have a huge impact on the English learning process. The key to the integration of English education resources is the storage of huge amount of English teaching data. Applying the technology and methods of cloud storage to the construction of English education resource integration can effectively save the educational resources of schools, improve the utilization rate of English education resources, and thus enhance the teaching level of English subjects. In this work, we examine the existing state of English education resource building and teaching administration and offer a way for creating a “private cloud” of English education materials. We not only examined the architecture and three-layer modules of cloud computing in depth, but we also analyzed the “private cloud” technology and built the cloud structure of English teaching materials on this foundation. We hope that this paper can help and inspire us to solve the problems of uneven distribution, irregular management, and difficult sharing in the construction of English education resources.

## 1. Introduction

With the continuous development of Internet of Things (IoT) technology and its educational application research, the promotion of IoT technology for educational management and educational teaching is becoming more and more obvious, and the popularization of IoT educational applications seems to be an inevitable trend [1]. The new IoT education application mode with education resource library as the core can greatly reduce the cost and technical threshold of IoT education application and make the popularization of IoT education application possible [2]. At present, various network educational resources, mainly network storage resources and educational resources that can be accessed through the net network, including various materials, multimedia courseware, integrity training videos, and e-books, are intended to provide support for teachers and students' use [3].

Traditional online English education resource platforms have many problems such as uneven distribution, irregular management, duplicate construction, difficulty in sharing, limited by storage capacity, and low security [4]. This makes it difficult for users to tap a large number of high-quality digital English education resources in the process of using them, and they are prone to low accuracy in information retrieval and low utilization of personalized resources [5]. However, the construction of English education resources is not a one-time performance completion, but a long-term process that must have long-term planning for sustainable development [6]. To eliminate the conventional closed model, data silos, and open up the environment for exchanging educational resources, it is required to regularly update and adapt construction methodologies [7]. In addition, the construction of educational resources must take service teaching as the main goal, and the basic principles of integrated planning, clear division of labor, broadening mode, strengthening application, and continuous innovation should be done in the construction process [8]. The existing resources need to be organized in a reasonable order and sorted out, while continuously introducing the latest and foreign excellent achievements [9].

RETRACTED

The purpose of using cloud computing to build an English education resource store is to serve many users at the same time [10]. The cloud computing system uses many technologies, among which virtualization, data storage, and cloud computing platform management are the most critical [11]. The cloud computing system uses redundant storage to ensure the reliability of data, and the distributed storage method can effectively store data [12]. The construction of an open English education resource platform based on cloud computing provides an important opportunity for the sharing of English education resources [13], and the basic architecture of cloud computing is shown in Figure 1. The feasibility analysis is as follows:

1. Expand the sharing of English education resources, avoid duplication of resources, and effectively improve the utilization of infrastructure. Since cloud computing supports crossplatform IoT terminal devices, the network can be used to share resources anytime and anywhere
2. Improving educational resource management. Through distributed and parallel computing, cloud computing analyzes and manages English education resources and stores and calculates them, and the high reliability can ensure the efficient operation of the open education resource platform

The goal of this study is to construct a “private cloud” environment and use cloud computing, a new Internet of Things technology, to overcome the shortcomings of the traditional English education resource platform. By establishing a large digital education platform for resource management and sharing, educational resources can be widely used. It can also serve as a reference for the development of cloud computing model education reform and information technology for English education.

RETRACTED

The paper's organization paragraph is as follows: the related work is presented in Section 2.  Section 3 analyzes the architecture of the cloud platform.  Section 4, discusses the design of English education resource storage system based on Eucalyptus private cloud platform. Finally, in Section 5, the research work is concluded.

## 2. Related Work

In this section, we define the analysis of the current situation of English online education resources, obstacles encountered in the construction of English online educational resources, and advantages of private cloud-based English education resource construction in detail.

### 2.1. Analysis of the Current Situation of English Online Education Resources

#### 2.1.1. Analysis of Resource Management Model of Network Education on Various Platforms

In terms of the current management modes of various English education resource repositories [14], they can be basically summarized into three types: centralized management, open management, and centralized plus open management. Centralized management emphasizes privacy and copyright protection [15], orderliness, and standardized use of educational resources to ensure security and effective use. With this approach, a single department is usually solely responsible for unified management. The model emphasizes that the characteristics of educational resources should fully reflect the professional advantages of each educational platform with distinctive cultural advantages. The disadvantage of this model, on the other hand, is the closed lack of openness. Because educational resources are often restricted to use within a single specific group, this greatly limits the space for utilization, is not conducive to fully reflecting their value, and is poorly shared. In the open management model, the idea is to open up. This management paradigm assigns different permissions to distinct groups of resource users and creates a security hierarchy for educational resources, allowing some users to have administrator privileges and upload resources. The advantage of open and interactive management is that users and managers can interact and by doing so, information resources can be continuously improved to a higher and higher level. It can truly reflect the needs of the users, and the resource effectiveness is fully reflected. The centralized management mode, together with completely open management, effectively avoids the disadvantages of both. Realizing openness in centralization and centralization in openness is the future development direction of education resource management model.

RETRACTED

#### 2.1.2. Current Situation of the Development of English Online Education Resources on Various Platforms

At present, the main form of network education resource construction is resource library [16]. From the construction of English education resource library of each platform, all of them have purchased online education resource library and online teaching platform [17]. Teachers, professionals, and software companies work together to integrate educational resources; conduct online courses, online teaching, and online course development; and build “high-quality courses.” From the perspective of the construction mode, there are mainly the following modes: (1) there are many companies engaged in research work in this area, they have made a large number of highly targeted teaching materials, direct purchase can save a lot of development costs in terms of manpower and financial resources, and these materials can be widely adapted to the majority of teachers' requirements; (2) resource sharing with various professional open websites; and (3) mainly for each platform's own teaching philosophy and the needs of teaching teachers.

### 2.2. Obstacles Encountered in the Construction of English Online Educational Resources

According to the survey of educational resource libraries on various platforms, it is found that many inventories have problems in the following aspects.

1. Resource construction emphasizes quantity but neglects quality

Today's educational resource repositories range from tens of GB to several TB. The platforms often store large amounts of data with large storage capacity. Platforms often take the large data of storage capacity as a selling point and spend a lot of effort to collect more resources without paying attention to the quality of resources, resulting in impractical resource contents that do not meet the needs of teaching and learning, reducing the availability of resources and leading to the waste of resources.

(2) Poor communication and interactive performance among users

The lack of communication between users and resource builders results in poor initiative of users, which prevents resource builders from getting timely feedback information. Because of the lack of systematic research and study to fully understand the needs of teachers and students in terms of usage, the dimension and depth of cooperation between resource builders and subject teachers are insufficient. The bearers of resource construction are often prone to work behind closed doors, measuring the effectiveness of resources by their own standards of take and take, thus causing the repository to frequently fail to find the needed resources and frustrating the motivation of teachers and students to continue using them.

(3) The efficiency and accuracy of educational resource retrieval is poor

The reason for this is mainly that the attribute labeling of resources is not rich and standard enough when data are stored. With the existing resources, it is too simple to provide query functions; it should provide a variety of query methods, such as keyword search, categorized information, combined query, tree view, search, and personalized full-text search.

RETRACTED

### 2.3. Advantages of Private Cloud-Based English Education Resource Construction

Cloud computing services were applied to all areas of English platform education resource construction by building a private cloud environment inside the platform to facilitate the completion of daily teaching activities and provide an efficient and stable education resource application environment for teachers and students [18]. Building cloud-assisted teaching is a new concept that involves several disciplines, and its main research includes theories of cloud computing on traditional educational resources and various factors that affect the application of educational exploration teaching methods, cloud computing, etc. [19]. It also includes the use of information technology to create and manage current educational resources, as well as the creation of new resource sharing models to ensure that educational resources are used to their full potential [20].

Private cloud education resource platform has the following advantages.

1. Cost reduction

The English education resource platform built by applying cloud computing network can effectively control the demand for hardware and the resulting costs. In traditional servers providing network services, we often encounter various hardware failures caused by hard disk damage brought about by long-term use of the server, which may lead to data loss and bring us irreparable damage. With a server using cloud storage, such problems can be avoided. We store data in a unified cloud file, and file reads are done in the cloud. Since in cloud computing clusters, the hardware requirements for server equipment are not high, old equipment can be reused without the need to buy high-grade new equipment. Even various old inexpensive PCs can be incorporated into the cloud storage system. In this way, the procurement cost of each platform is reduced, while the service life of the hardware is greatly improved. In addition, virtualization technology can be used to consolidate the school's original group of server machines into a powerful cloud cluster through the configuration of virtualization software, which allows the school to save a lot of money in terms of hardware expenses and maintenance, etc.

(2) Easy sharing of resources

Working together and sharing resources, solving problems, and using resources in a virtual organization to fulfil the new needs of users are another significant element of cloud computing. Cloud computing is an integrated computing system in which users in a private cloud can share the same environment and access their desired resources at any time and from any location. At the same time, information and resources can be shared by writing a number of different computer applications that are based on the characteristics of cloud computing and allow users to access them independently for extensive collaborative learning through cooperation.

(3) Security

While cloud computing can improve business agility and efficiency, it can also introduce new risks and threats. Cloud users will face unprecedented challenges, not only in terms of technology, but also in terms of making significant changes in the process. Yet, a cloud-based English education resource platform eliminates the need to consider the current common security concerns regarding cloud computing in addition to the security issues common in traditional online education. On the one hand, because the cloud computing education platform is used by a single group, it is easy to implement regulatory control for users in the cloud platform. On the other hand, the architecture and design of the cloud platform also fully consider the security policy and other related issues. In addition, the cloud platform uses user authentication and access control to control the security risks of each layer.

RETRACTED

## 3. Architecture of the Cloud Platform

In this chapter, we define the private clouds, private cloud platform based on Eucalyptus infrastructure, Hadoop-based massive data storage platform, and HBase in depth.

### 3.1. Private Clouds

Private clouds are clouds for your own internal use and are deployed within the firewall of the English education platform's data center. Since it is built for the platform's separate use, it can effectively control data security and data quality in the private cloud. Based on the existing facilities, the platform can adopt the private cloud construction mode and deployment method that meet its own needs and combine the characteristics of cloud computing, as shown in Figure 2 for the private cloud deployment schematic.

The private cloud is deployed behind the user's firewall and is connected to the outside Internet via routing and firewall. Inside the firewall, the private cloud provides various cloud services to the IoT endpoints below. Private clouds have similar functionality to public cloud platforms, with common private cloud platforms such as IBM CloudBurst and Microsoft Windows Azure. A common private cloud architecture is shown in Figure 3.

From Figure 3, we see that the private cloud contains the following management platforms:

1. Resource management: computing, storage, network resources, applications, and operation (use) interface calls to achieve the management and monitoring of resources
2. Network management system: through the network management interface, used to receive a variety of information network management, including network configuration, network performance, and alarm information
3. Operation management: the private cloud operation management platform sends messages to users or operation managers
4. System management: the unified identity authentication method of single sign-on is used to enter the system management

Users can apply for and use resources through the private cloud platform, and operation managers can complete operation management operations for users and resources through the operation management portal of the private cloud operation management platform.

### 3.2. Private Cloud Platform Based on Eucalyptus Infrastructure

Eucalyptus is divided into five main parts, which collaborate with each other to provide services. They are Cloud Controller (CLC), Cluster Controller (CC), Node Controller (NC), Walrus Storage Controller, and Storage Controller (SC). Various components of Eucalyptus for flexible configuration of various topology administrators adjust the cloud platform configuration. Different levels of security are considered to meet security and management needs. Eucalyptus can topologize one and multiple clusters. A single cluster requires at least two servers: a CC, SC, and CLC, and other small NCs; this configuration is mainly used for testing. In a multicluster deployment, different components (CC, SC, and NC) can be set to different machines. If it is used for a large number of calculations, a multicluster configuration is most suitable. As demonstrated in Figure 4, resource allocation may be done across zones and nodes, and a node failure does not affect the entire cluster, leading to high availability, load balancing, and resource distribution among clusters to handle enormous data processing tasks.

### 3.3. Hadoop-Based Massive Data Storage Platform

Hadoop is a distributed system infrastructure in which users develop applications without the need to understand the detailed information system mastery. In Hadoop distributed applications, users can take full advantage of high-speed computing clusters and storage capabilities without having to understand the detailed information system mastery. HDFS is short for Hadoop's file system. HDFS is highly fault-tolerant, can be used on low-cost hardware, and has high access rates to applications. It can be used on low-cost hardware and has a high access rate to applications, making it suitable for applications with large amounts of data to compute.

RETRACTED

HDFS, a distributed file system for use on general purpose hardware devices, is part of the composition and design of Nutch's search engine project under Hadoop. HDFS uses a master-slave architecture and is more like a hierarchical file system from the user's perspective. File commands to create, delete, move, or rename can be performed. Due to its own characteristics, HDFS is architected as a series of specific nodes. These nodes include a NameNode that provides metadata services and a series of DataNodes that provide storage blocks to accommodate applications with large data sets, as shown in Figure 5.

The files stored in HDFS are divided into 64 M-sized chunks, which are then copied to multiple data nodes. The NameNode controls all file operations in HDFS, and all communication within HDFS uses the standard TCP/IP protocol.

#### 3.3.1. NameNode

In Hadoop, the NameNode is the software that runs on the computer. The NameNode is the master server, responsible for managing files and namespaces, accessing clients, and the administrator of the entire system. The NameNode determines whether data files are replicated to the DataNode.

The HDFS cluster has only one NameNode, thus simplifying the overall architecture of the system Hadoop, which manages all the metadata of the file system. The functions are composed of the following points:

1. The data NameNode in HDFS is used to maintain file system metadata, such as names, spaces, and data exchange information for data block mapping. It is also responsible for managing client access to files, such as opening files or directories, closing, and renaming
2. Detecting NameNode periodically collects the load on this DataNode node, during which the DataNode may lose contact with NameNode due to failure. If a heartbeat packet is lost, the lost DataNode is marked as failed and no new I/O requests are sent to them, while all data within this node will be cleared
3. Namespace management NameNode manages the system namespace. Any changes to the generated data are logged by the NameNode using EditLog. Also, the entire system uses FsImage for storage. NameNode stores the file system in the FsImage and logs it inside EditLog
4. Listening and processing requests to the client DataNode give NameNode the responsibility to monitor and process the requests. Based on the request, it reads and writes files, deletes them, and performs other file operations

RETRACTED

#### 3.3.2. DataNode

Each node of a DataNode deployment Hadoop cluster is a Hadoop instance, usually a piece of software running on a machine. A file is usually divided into several chunks of data, and one of the DataNode nodes is responsible for managing its own data storage and reading client requests. The DataNode receives read and write client requests and, together with the NameNode, creates, deletes, and copies blocks of data. The functions of the data nodes are summarized as follows:

1. Copy data

First, the file system server process on the client side gets a list of the blocks of data being copied from the NameNode, then copies the file blocks cached by the client to the first DataNode node, and simultaneously transfers that part to the second DataNode node. This is repeated until the copy of the file block and its data block is completed.

(2) Read and write data blocks

By contacting the client file system in the service process, when it receives a request for work from the client file system, the DataNode starts interacting with the NameNode to determine the need to create file blocks, delete, and copy, and after receiving permission from the NameNode, the DataNode client on the DataNode specified by the file system performs the specified operation.

(3) Send a heartbeat message and a block report to the NameNode

Each DataNode sends a message and file status report block to the NameNode periodically to determine the status of those DataNodes based on that report. In addition, the DataNode starts, begins scanning the local file system, and creates a list of all HDFS blocks, then sends a report to the NameNode.

### 3.4. HBase

HBase is an open-source distributed database storage schema, which also belongs to the Apache Hadoop project subproject. It is a highly reliable, high-performance, scalable, and powerful database system that can be built on servers that use it for the overall structure of a large data storage cluster. As shown in Figure 6, the HBase file storage system is Hadoop HDFS. Hadoop MapReduce is used to handle the massive data computation in HBase. Zookeeper is a unified scheduling collaboration service.

## 4. Design of English Education Resource Storage System Based on Eucalyptus Private Cloud Platform

In this section, we define the infrastructure layer design, platform service layer design, software service layer design, and database design in detail.

We share resources and enhance interaction for collaborative learning, and under the concept of computer-assisted teaching, this led to the design of a private cloud-based English education resource storage platform. The design idea not only integrates the theoretical research but also reflects the idea of preparation stage, and its overall architecture is shown in Figure 7.

RETRACTED

### 4.1. Design of Functional Submodules of Private Cloud-Based English Education Resource Storage Platform

#### 4.1.1. Infrastructure Layer Design

The core technologies of the private cloud-based English education resource storage platform involve virtualization technology, data storage and management, device maintenance, redevelopment technology, and load balancing. Virtualization technology not only refers to the virtualization of applications but also can refer to the virtualization of hardware devices. In the infrastructure service layer, virtualization technology can set various resources into a virtual resource pool and complete the unified management maintenance and scheduling of resources. Users do not need to know and manage the devices in the infrastructure service layer, and they can just arrange the storage devices and install the operating system and client software according to their needs. The education resource sharing platform can scale and adjust the resources well by using the technology of virtualization, which provides a strong technical support for the dynamic management of cloud computing resources. The infrastructure service layer is shown in Figure 8.

### 4.2. Platform Service Layer Design

In the field of education and teaching, the service layer of the PaaS platform built is based on the cloud storage feature of educational resources. On this platform, cloud services integrating development, testing, and operation are provided for education practitioners, educational institutions, or enterprises. The PaaS platform service layer also includes the environment needed for developing the teaching resource cloud platform, such as development, testing, operation, and maintenance. The PaaS platform service layer also formulates standard Web protocols, data formats, SDKs, and APIs and encapsulates common functions into header files for developers to call, which greatly reduces the development cycle and difficulty of enterprises, facilitates future maintenance, and improves the utilization of educational resources. It also improves the utilization of educational resources. In the private cloud-based English education resource storage solution introduced in this paper, the architecture diagram of PaaS is given in Figure 9.

According to the given PaaS architecture diagram, PaaS is mainly composed of two parts, which are the base platform and the service platform. The base platform generally provides environmental support for the development of application service software, such as performance management, storage management and computing, system billing, and forensic management and grid computing services, which are not visible to users. The service platform is mainly for user use and provides the environment required for application development, including development, testing, and running environments. During application development, both offline and online situations are supported. When the application is running, PaaS is in a hosted state and also features online automatic loading of the latest version of the application, real-time tracking, and traffic calculation.

RETRACTED

### 4.3. Software Service Layer Design

The software service layer is a direct user-oriented platform on the configured education resource sharing platform. Users directly access resources, share resources, store resources, etc. after logging in through the login interface. The software service layer is user-oriented, and the user's perception and experience of using it are directly reflected in the application service, which is called the value source of the cloud platform client, where all the data and information of educational resources are stored, directly facing the user.

#### 4.3.1. Educational Resource Production System Design

Aiming at the current problems of unreasonable information deployment, poor system operation, and poor human resource interactivity in the educational resource production system, the private cloud-based educational resource storage solution proposed in this paper can solve these problems well. By building a private cloud-based educational resource storage sharing platform, teachers and students can access a huge amount of teaching resources, which is convenient not only for teachers to teach production classes and assign after-class homework but also for students to finish their homework on time and submit it to teachers for review. In this cloud platform, students can also study according to their own needs and can leave messages with their teachers about their confusion after studying, which strengthens the interaction between teachers and students and also helps teachers to better understand students and help them learn. At the same time, in order to build the educational resource system, three subsystems are given according to the classification of students' needs, which are courseware production, assessment, and management.

1. Courseware production subsystem

The courseware production subsystem is mainly to provide convenient services for teaching staff, and it is a key part of the education resource cloud platform. There are various resources such as text, photos, audio files, and video files distributed on the network. Teachers can integrate these resources through the education resource sharing platform and make an editable teaching file and then share this file on the education cloud platform for everyone's reference and learning.

(2) Assessment subsystem

Because it is mainly for the pedagogue, the assessment subsystem is mainly to help teachers better assign homework and help students better complete their homework, and most importantly, teachers can see the homework in time after students finish it and also can review and interact online.

(3) Educational resource management subsystem

The management subsystem is mainly responsible for the management and maintenance of the system. The system management includes the registration of new users and the permissions of student users and teacher users. In this system, users are allowed to share their own resources on the platform, and other users can access and study them.  Figure 10 shows the infrastructure diagram of the educational resource management subsystem.

RETRACTED

As can be seen from Figure 10, the management subsystem contains four modules, each of which implements a different function. Four databases with varied functionalities are also set up, with the main purpose of storing various types of data. The management subsystem's registration module performs resource verification, checks that there are no issues, and then determines it to be lawful before saving it in the database. At the same time, some annotated information about the resources will be stored in the registration database, which is convenient for the search module. The access control module is mainly to complete user verification, and those who pass the verification are normal users before they can manage the data resources. In the face of massive data, the cache module can exponentially improve the rate and accuracy of resource screening. The function of the synchronization module is to complete the mirror registration database and the cloud platform data information comparison.

### 4.4. Database Design

The information stored on the server of the English education resource cloud platform is mainly the information of network nodes, the information of materials uploaded by users, and some basic information filled in by users when they register. The following describes the design of database keywords involved in the education cloud platform.  Table 1 is the user information table for the initially registered users; when there is a newly registered user, it is to be filled out according to the table information, mainly concerning the user name, password, and user rights.  Table 2 is the user information table; this table is mainly used to store the user's private information, including birthday, home address, and hobbies.  Table 3 is the resource table; this table stores the user's resource information, which involves whether the information is public or not, the type of information, etc.

RETRACTED

## 5. Conclusion

Cloud storage technology and methodologies are being utilized to integrate English education resources as an emerging concept, which can significantly improve the usage rate of online platform English education resources and teaching efficiency. We provide a private cloud storage platform for English educational resources, combining cloud computing technologies, analyzing its architecture and execution, and implementing data transmission and storage using the Hadoop platform. The implementation of this platform is based on the existing mature cloud platform application examples and requires the synergy between various technologies such as multitenancy, distributed computing, and virtualization to build a cloud service platform for English education resource storage. This solution may open up new possibilities for the creation and distribution of English educational content.

## Figures and Tables

**Figure 1:** Cloud computing architecture.

**Figure 2:** Private cloud deployment schematic.

**Figure 3:** Private cloud architecture.

**Figure 4:** Eucalyptus single and multicluster topologies.

**Figure 5:** Simplified view of an HDFS cluster.

**Figure 6:** Hadoop system architecture.

**Figure 7:** The architecture of English education resource storage platform in private cloud.

**Figure 8:** English education resource storage infrastructure service layer.

**Figure 9:** Education resource storage platform PaaS layer architecture diagram.

**Figure 10:** Educational resource management subsystem structure diagram.

**Table 1:** User table.

Field	Type	Null	Default	Comments	MIME
id	Int (128)	No		Primary key	
User_name	Varchar (128)	No		User name	
Password	Varchar (128)	No		User password	
Priority	Tinyint (10)	Yes	NULL	User rights	

**Table 2:** User information form.

Field	Type	Null	Default	MIME
id	Int (8)	No		
User_id	Int (8)	No		
User_emai1	Varchar (40)	No		
User_name	Varchar (40)	Yes	Null	
User_address	Varchar (120)	Yes	Null	
User_sex	Varchar (4)	Yes	Null	
User_birthday	Varchar (20)	Yes	Null	
User_intro	Varchar (400)	Yes	Null	
User_time	Timestamp	No	Current_timestamp	
User_profession	Varchar (200)	Yes	Null	
User_labe1	Varchar (200)	Yes	Null	

**Table 3:** User resource table.

Field	Type	Null	Default	MIME
id	Int (11)	No		
User_id	Int (11)	No		
Resource_name	Varchar (128)	Yes	Null	
Resource_info	Text	Yes	Null	
Resource_type	Varchar (11)	Yes	Null	
Resource_grade	Varchar (11)	Yes	Null	
Resource_address	Varchar (128)	Yes	Null	
Resource_version	Varchar (64)	Yes	Null	
Resource_pub_se1	Varchar (11)	No	Null	
Resource_suit	Varchar (20)	Yes	Null	
Resource_discip1ine	Varchar (20)	Yes	Null	
Resource_edition	Varchar (20)	Yes	Null	
Resource_specia1	Varchar (20)	Yes	Null	
Resource_a11ow_down1oad	Tinyint (1)	Yes	Null	
Resource_regi	Timestamp	No	Current_timestamp	
Resource_update	Timestamp	No	0000-00-00 00:00:00	

RETRACTED

## Data Availability

The datasets used during the current study are available from the corresponding author on reasonable request.
